# Proliferation in culture of primordial germ cells derived from embryonic stem cell: induction by retinoic acid

**DOI:** 10.1042/BSR20160441

**Published:** 2016-12-23

**Authors:** Zohreh Makoolati, Mansoureh Movahedin, Mehdi Forouzandeh-Moghadam

**Affiliations:** * Department of Anatomical Sciences, Faculty of Medicine, Fasa University of Medical Sciences, Fasa 74616-86688, Iran; † Department of Anatomical Sciences, Faculty of Medical Sciences, Tarbiat Modares University, Tehran 14115-175, Iran; ‡ Department of Biotechnology, Faculty of Medical Sciences, Tarbiat Modares University, Tehran 14115-175, Iran

**Keywords:** embryonic stem cell, primordial germ cell, proliferation, retinoic acid

## Abstract

An *in vitro* system that supports primordial germ cells (PGCs) survival and proliferation is useful for enhancement of these cells and efficient transplantation in infertility disorders. One approach is cultivation of PGCs under proper conditions that allow self-renewal and proliferation of PGCs. For this purpose, we compared the effects of different concentrations of retinoic acid (RA), and the effect of PGCs co-culture (Co-C) with SIM mouse embryo-derived thioguanine- and ouabain-resistant (STO) cells on the proliferation of embryonic stem cells (ESCs)-derived PGCs. One-day-old embryoid body (EB) was cultured for 4 days in simple culture system in the presence of 5 ng/ml bone morphogenetic protein-4 (BMP4) (SCB group) for PGC induction. For PGC enrichment, ESCs-derived germ cells were cultured for 7 days in the presence of different doses (0–5  μM) of RA, both in the simple and STO Co-C systems. At the end of the culture period, viability and proliferation rates were assessed and expression of mouse vasa homologue (Mvh),  α6 integrin,  β1 integrin, stimulated by retinoic acid 8 (Stra8) and piwi (Drosophila)-like 2 (Piwil2) was evaluated using quantitative PCR. Also, the inductive effects were investigated immunocytochemically with Mvh and cadherin1 (CDH1) on the selected groups. Immunocytochemistry/PCR results showed higher expression of Mvh, the PGC-specific marker, in 3  μM RA concentrations on the top of the STO feeder layer. Meanwhile, assessment of the *Stra8* mRNA and CDH1 protein, the specific makers for spermatogonia, showed no significant differences between groups. Based on the results, it seems that in the presence of 3 μM RA on top of the STO feeder layer cells, the majority of the cells transdifferentiated into germ cells were PGCs.

## INTRODUCTION

Primordial germ cells (PGCs), the progenitors of spermatogonia and oogonia, are the bridges between stem cells and gametes. These cells are a highly specialized cell population that arises from the epiblast and are requisite for the maintenance of the species [1]. There are three critical phases during the life cycle of PGCs: specialization, migration/proliferation and eventually pre- and postnatal sex-specific development. Common signals important for germ cell specification in epiblast are found in mammals [2,3]. Several groups showed that bone morphogenetic protein-4 (BMP4), members of the transforming growth factor beta (TGF-b) family of signalling molecules, was specifically required for germ cell differentiation in mice [4–12].

During the second phase of germ cell development, the PGCs migrate from the base of the allantois to the genital ridge and proliferate in this way. PGCs have a limited period of proliferation *in vitro* and then go into growth arrest, which is similar to their developmental changes *in vivo*. It is important to achieve enough PGCs to produce the gametes *in vitro*. Nakatsuji and Chuma [13] have found that in the presence of multiple growth signals, PGCs can restart rapid proliferation. Several culture systems for viability and proliferation of PGCs have been established up to now. These systems include: adding chicken stem cell factor (chSCF) and fibroblast growth factor 2 (FGF2) to PGC lines [14], addition of retinoic acid (RA) to PGC-like cells differentiated from mouse skin-derived stem cells [15], using steel factor (SLF) and leukaemia inhibitory factor (LIF) [16–19], tumour necrosis factor (TNF)-α [20], RA [21], buffalo rat liver cells (BRL-CM) [22], forskolin (FK), macrophage growth factor (MGF) and kit ligand (KL) [20] in the culture of PGCs derived from epiblast and genital ridge, co-culture (Co-C) of epiblast-derived PGCs with feeder cell monolayer Sertoli cells or SIM mouse embryo-derived thioguanine- and ouabain-resistant (STO) [16,19,23] and using combination of FK, KL and fibroblast feeder cells in culture of human PGCs derived from genital ridge [24–26].

RA is a vitamin A-derived, small non-peptidic lipophilic molecule that binds to nuclear RA receptor and has the ability to stimulate meiosis in both sexes [27–29].

So far, however, there has been little discussion about the role of RA on PGC proliferation [21,30]. Koshimizu et al. [21] observed stimulation of mitotic activity by RA treatment at all stages of PGC examined (8.5, 11.5 and 13.5 days postcoitum). Morita and Tilly [30] have reported the mitogen activity of RA for germ cells during *in vitro* foetal mouse oogenesis. Also, the role of RA in inducing PGC formation from 3 to 9 days old mouse embryoid bodies (EBs) [31], skin-derived stem cells [15] and chicken genital ridge [32] was reported.

However, the role of RA on the proliferation of PGCs differentiated from embryonic stem cells (ESCs) has not been studied. The aim of the present study was to find more optimal culture conditions for proliferation of PGCs derived from mouse ESCs *in vitro*. For this purpose, we examined the efficacy of both STO Co-C system and RA, in inducing proliferation of ESCs-derived PGCs.

## EXPERIMENTAL

### Cell culture medium

CCE mouse ESCs established from 129/Sv mouse strain (a kind gift from Dr John Draper, Centre for Stem Cell Biology, Sheffield University, U.K.) were cultured in Dulbecco's modified Eagle's medium (DMEM) with high glucose, pyruvate and L-glutamine (Gibco) with 20% FBS (Gibco), 0.1 mM non-essential amino acids (Sigma–Aldrich), 0.1 mM β-mercaptoethanol (Sigma–Aldrich), 3.7 g/l NaHCO_3_ (Sigma–Aldrich), 100 units/ml penicillin, 100 μg/ml streptomycin (Gibco) and 1000 units/ml LIF (Sigma–Aldrich). Undifferentiated ESCs were cultured at 37°C, 5% CO_2_ and 95% humidity, and medium was renewed daily. The present work is approved by Ethical Committee of Tarbiat Modares University.

### Passage of mouse embryonic stem cells

Undifferentiated ESCs were passaged every 2 days by trypsin (0.25%; Merck)/EDTA (1 mM; Sigma–Aldrich) dissociation. For passaging, medium was aspirated, dishes were rinsed with PBS and trypsin–EDTA was added enough to cover the surface of the tissue culture dish. After incubation at room temperature (20°C) and lift-off cells from the plate, pipetting was done and 15% FBS in DMEM was added to inhibit trypsin–EDTA. The cell suspension was centrifuged at 200 ***g*** for 8 min at room temperature and the cells were split on to new tissue culture dishes.

### Embryoid body formation and induction protocol

CCE mouse ESCs were trypsinized and 2  × 10^5^ cells seeded in six-well culture plates. The cells incubated for 24 h in DMEM medium containing 20% FBS and LIF was removed. After 1 day, EBs were trypsinized, counted and replated on to a 96-well microplate (8×10^4^cells in each well) for continuation of the induction protocol. In the initial stage, BMP4 was added at concentration of 5 ng/ml for 4 days to induce PGC differentiation [10]. In the next stage, the cells were treated for 7 days with different doses (0–5 μM) of RA both in the simple and STO Co-C systems for PGC enrichment. In Co-C system, as confluency of the STO cells reached approximately 90%, the cells treated with 10 μg/ml mitomycin C (Sigma–Aldrich) for 2 h and washed with PBS for 3 to 4 times. After that, BMP4-treated cells were transferred into Millicell 24-well cell culture insert plates and co-cultured with mitomycin-treated STO cells.

### Assessment of proliferation rate and viability percentage

The cells in the STO Co-C system both in the presence or absence of 0–5 μM concentrations of RA were harvested, prepared as a single-cell suspension and stained with 0.4% Trypan Blue (Sigma–Aldrich). Counting was done using a haemocytometer. The mean number of whole cells and living cells were considered as proliferation rate and viability percentage respectively.

### RNA extraction and reverse transcription

Total RNA from simple culture system with BMP4 (SCB), simple culture system with different doses of RA (0–5 μM) and STO Co-C system with different doses of RA (0–5 μM RA + Co-C) groups and whole testis as a positive control was extracted using the RNX-Plus™ kit (CinnaGen) according to the following protocol. Approximately 3×10 homogenized cells or 50–100 mg of testis tissues were incubated with 1 ml of RNX-Plus solution for 5 min at room temperature. After adding chloroform, solution was centrifuged at 12000 ***g*** for 15 min at 4°C. The upper phase was conveyed to another tube, an equal volume of propan-2-ol was added and the mixture was centrifuged at 12000 ***g*** for 15 min. The resulting pellet was washed with 70% ethanol and dissolved in diethylpyrocarbonate (DEPC)-treated water. The purity and integrity of the extracted RNAs was determined using UV spectrophotometer (DPI-1, Kiagen). Before cDNA synthesis, the extracted RNA was treated with DNase I using Fermentas kit for removal of genomic contamination.

The cDNA synthesis reaction was done by RevertAid™ First strand cDNA Synthesis Kit (Fermentas) with the use of oligo(dT) primers. Briefly, 1 μg of total RNA was reverse transcribed with 20 units/μl RNase inhibitor (RNasin), 1 mM dNTP, 2.5 ml of 10× PCR buffer, 0.5 μg oligo(dT) and 200 units of RevertAid™ M-MuLV reverse transcriptase (Fermentas) in a 20 μl reaction. The samples were placed in a thermocycler (Bio–Rad Laboratories) for 60 min at 42°C and for 10 min at 70°C afterwards.

### Quantitative real-time PCR (RT-qPCR)

In order to verify the reaction conditions, optimization procedures for annealing temperatures of the primers and specific products were done before PCR reaction. PCR was carried out with gene specific primers (Table 1) on Rotor-Gene 3000 thermocycler (Corbett Life Science) using PCR master mix (CinnaGen) and SYBR Green I (Fluka). The PCR conditions were: an initial melting cycle, 4 min at 94°C to activate the polymerase, followed by 40 cycles (94°C for 20 s, 57°C for 30 s and 72°C for 30 s). After completing each PCR run, melt curve analysis was used to confirm the amplified product. Efficiency was determined for each gene using standard curve obtained with the logarithmic dilution series of testis cDNA over a 10-fold range. The comparative *C*_T_ (cycle threshold) method of Pfaffl was used to determine the ratio of gene expression [33]. In SCB group, target genes expression was normalized to reference gene (β2m). However, in 0–5  μM RA and 0–5 μM RA+Co-C groups, gene target gene/housekeeping gene (β-actin) were calculated, calibrated to the before stage (SCB group) and compared with the different groups. In all reactions, mouse testis was used as positive control.

**Table 1:** Primer sequences, accession numbers, expected product size and melting temperatures of germ cell and housekeeping genes

Accession number	Gene	Primer (Forward/Reverse)	Product size (bp)	Product melting temperature (°C)	Reference
NM_001145885	*Mvh*	5′-GCTCAAACAGGGTCTGGGAAG-3′/5′-GGTTGATCAGTTCTCGAG-3′	145	74.2	(Toyooka et al. 2003)
NM_009292	*Stra8*	5′-TCACAGCCTCAAAGTGGCAGG-3′/5′-GCAACAGAGTGGAGGAGGAGT-3′	441	77.4	(Makoolati et al. 2011)
NM_008397	*α6 integrin*	5′-GAGGAATATTCCAAACTGAACTAC-3′/5′-GGAATGCTGTCATCGTACCTAGAG-3′	398	77.2	(Cooper, Tamura et al. 1991)
NM_010578	*β1 integrin*	5′-GTGACCCATTGCAAGGAGAAGGA-3′/5′-GTCATGAATTATCATTAAAAGTTTCCA-3′	217	75.2	(Holers, Ruff et al. 1989; Holers et al. 1989)
NM_021308	*Piwil2*	5′-GCACAGTCCACGTGGTGGAAA -3′/5′-TCCATAGTCAGGACCGGAGGG-3′	681	81.8	(Lee et al. 2006)
NM_009735	*β_2_m*	5′-TGACCGGCCTGTATGCTATC-3′/5′-CACATGTCTCGATCCCAGTAG-3′	316	77.6	(Boroujeni, Salehnia et al. 2008)
NM_001101	*β-actin*	5′-TCCCTGGAGAAGAGCTACG-3′/5′-GTAGTTTCGTGGATGCCACA-3′	131	79.2	(Wu, Tsai et al. 2011)

### Immunocytochemistry for Mvh (VASA, Ddx4) and CDH1

The immunocytochemical evaluation was done in the following groups: SCB, STO Co-C and 3 μM RA+Co-C. Approximately 5 h prior to immunostaining, clumps of cells were trypsinized and resuspended in 96-well microplate. Adherent cells were fixed in 4% paraformaldehyde for 20 min at room temperature. Fixed cultured cells were rinsed in PBS, incubated in HCl (2 M) at room temperature for 30 min and washed with borate buffer. Non-specific antibody reaction blocking was performed in 10% normal goat serum (Sigma–Aldrich). To permeabilize the cells, they were treated with 0.3% Triton X-100 (ICN) in PBS. Then, the specimens were incubated with 1/100 diluted cadherin1 (CDH1) (Calbiochem) and mouse vasa homologue (Mvh) (Abcam) antibodies overnight at 4°C. It was followed by incubation with 1/10 diluted secondary FITC goat anti-mouse IgG (RayBiotech) against CDH1 and goat anti-rabbit IgG antibody (RayBiotech) against Mvh for 2 h at room temperature. Finally, drying and mounting were performed. To determine the percentage of immunoreactive cells, the cells showing specific immunolabelling were estimated by counting a total of 100 cells at 400× with an inverted immunofluorescent microscope. In all immunostainings, a negative control was used by staining with secondary antibody only.

### Statistical analysis

Statistical analysis was done with SPSS 13.0 software. Data were shown as mean  ± S.D. and represent the average of three separate experiments. One-way ANOVA and Tukey's post-test were used to determine the statistical significance of observed differences in the level of *P*≤0.05.

## RESULTS

### Evaluation of proliferation rate and viability percentage

The proliferation rate and viability percentage of the RA-treated cells and their controls in all groups were determined using 0.4% Trypan Blue and are presented in Table 2. There was significant decrease in proliferation rates of the 3 and 5 μM RA and 0–5 μM RA  + Co-C groups relative to the 0 μM RA group (*P*<0.05). As shown in Table 2, the lowest rate of viability percentage was seen in 5 μM RA group that had significant differences with 0–2 μM RA and 2 μM RA+Co-C groups (*P*<0.05). Also, significant decrease in viability percentage of 4 μM RA group compared with the 1 μM RA group was observed (*P*≤0.05).

**Table 2:** The comparison (mean ± S.D.) between the mean of the proliferation rate and viability percentage of cells treated with different concentrations of RA in the presence or absence of STO Co-C feeder layer cells The primary cell number in all groups was equal to 3×10^5^. ashows significant difference with 0 μM RA, ^b^indicates significant difference with 5 μM RA and ^c^demonstrates significant difference with 1 μM RA group in the same columns (*P*≤0.05).

Group	Proliferation rate	Viability percentage
0 μM RA	2.32±2.1	74.34±0.75^b^
1 μM RA	1.65±1.8	79.9±1.1^b^
2 μM RA	1.36±0.75	70.83±1.2^b^
3 μM RA	0.19±0.5a	57.73±0.51
4 μM RA	0.63±1.2	48.35±0.45^c^
5 μM RA	0.15±1.8a	38±0.23
0 μM RA+Co-C	0.43±0.74a	64.27±0.87
1 μM RA+Co-C	−0.2±0.98a	65.79±1.4
2 μM RA+Co-C	0.17±0.56a	66.17±2.1^b^
3 μM RA+Co-C	−0.1±1.1a	63.54±1.5
4 μM RA+Co-C	0.04±0.43a	58.09±1.48
5 μM RA+Co-C	−0.07±1.3a	58.78±0.76

### Germ cell genes expression profiles

Quantitative PCR revealed variations in the expression of germ cell genes in different groups. Molecular results showed that the mean normalized expression of Mvh, α6 integrin, β1 integrin, stimulated by retinoic acid 8 (Stra8) and piwi (Drosophila)-like 2 (Piwil2) in SCB group were 6.7×10^−3^ ± 0.005, 0±0, 0.25±0.16, 4.2×10^−5^ ± 10^−6^ and 0.6±0.45 respectively (Figure 1).

**Figure 1:** Gene expression profiling analysis Ratio of genes expression in 0–5 μM RA concentrations and 0–5 μM RA concentrations+STO Co-C groups relative to simple culture with BMP4 (SCB) group. In the Mvh graph, ashows significant difference with 3 μM RA+STO Co-C and ^b^demonstrates significant difference with 5 μM RA+STO Co-C groups. In the α6 integrin chart, ashows significant difference with 0 μM RA, ^b^demonstrates significant difference with 0 μM RA+STO Co-C, ^c^indicates significant difference with 2 μM RA+STO Co-C and ^d^reveals significant difference with 5 μM RA+STO Co-C groups. In the β1 integrin diagram, ashows significant difference with other groups. In the Stra8 graph, ashows significant difference with 2 μM RA+STO Co-C and ^b^demonstrates significant difference with 5 μM RA+STO Co-C groups and in the Piwil2 chart, ashows significant difference with 4 μM RA, ^b^demonstrates significant difference with 0 μM RA+STO Co-C and ^c^indicates significant difference with 3 μM RA+STO Co-C groups (*P*<0.05).

The maximum and minimum expressions of Mvh, the PGC specific marker, were seen in the 3 and 5 μM RA+Co-C groups, in that order. The ratio of gene expression in 0–5 μM RA and 0–5 μM RA+Co-C groups relative to SCB group was 3.5-, 1.11-, 1-, 5.37-, 6.34-, 5.39-, 1.66-, 1.3-, 1.75-, 7.32-, 3.25- and 0.002-folds respectively. There were significant differences in Mvh expression among 3 μM RA+Co-C group both with SCB group and with 1 and 2 μM RA and 0, 1, 2 and 5 μM RA+Co-C groups (*P*<0.05, Figure 1).

The level of the α6 integrin gene expression was increased in the 0–5 μM RA and 0–5 μM RA+STO Co-C groups. The increased ratios of α6 integrin expression relative to SCB group were 29.4-, 19.83-, 18-, 59.55-, 6.85-, 7.15-, 45.33-, 11.5-, 69-, 6.5-, 8- and 63-folds in the 0–5 μM RA and 0–5 μM RA+Co-C groups respectively. The increased ratio of α6 integrin expression in the 2 and 5 μM RA+STO Co-C and in the 3 μM RA groups had statistical differences with other groups (*P*<0.05). Also, the increased expression in 0 μM RA+STO Co-C group shows significant difference with SCB, 4 and 5 μM RA, and 1, 3 and 4μM RA+STO Co-C groups (*P*<0.05, Figure 1).

The levels of β1 integrin mRNA in the 0–5 μM RA and 0–5 μM RA+Co-C groups relative to SCB group were 0.0018-, 0.0003-, 0.00004-, 0.0001-, 0.0001-, 0.0045-, 0.00009-, 4.5-, 0.0005-, 0.0008-, 0.0001- and 1.0001-folds respectively. The maximum expression of β1 integrin in the 1 μM RA+Co-C group was significantly different compared with the other groups (*P*<0.05, Figure 1).

Investigation of the *Stra8* gene, the late germ cell marker, showed increased level of this gene in the experimental groups compared with SCB group. The increased ratios of Stra8 expression relative to SCB group were 5.33-, 2.5-, 2.33-, 2.5-, 3.33-, 1.21-, 1.99-, 2.83-, 11.16-, 1.33-, 1.83- and 8.66-folds in 0–5 μM RA and 0–5 μM RA+Co-C groups respectively. Increased expression of Stra8 in 2 μM RA+Co-C group showed significant differences with SCB and all other groups of the study except 5 μM RA+Co-C group (*P*<0.05). Also, the increased level of *Stra8* mRNA expression in 5 μM RA+Co-C group was significantly different compared with the SCB and all groups excluding 0 μM RA group (*P*<0.05, Figure 1).

The level of *Piwil2* gene expression was increased in the all experimental groups relative to SCB group. The increased ratios of *Piwil2* in 0–5 μM RA and 0–5 μM RA+Co-C groups compared with the SCB group were 6-, 2.66-, 0.4-, 0.32-, 8.16-, 1.82-, 8.88-, 4-, 0.4-, 11.4-, 0.9- and 5.33-folds correspondingly. The maximum expression of Piwil2 in the 3 μM RA+Co-C group was significantly different compared with the other groups (*P*<0.05) except 4 μM RA group. Also, the increased ratio of Piwil2 in 0 μM RA+Co-C group was significantly different from SCB, 1–3 and 5 μM RA and 2 and 4 μM RA+Co-C groups (*P*<0.05). Similarly, significant increase was seen between the 4 μM RA group compared with the SCB, 2, 3 and 5 μM RA and 2 and 4 μM RA+Co-C groups (*P*<0.05, Figure 1).

### Immunocytochemistry for Mvh and CDH1

Based on the results of molecular studies, the 3 μM RA+Co-C group was selected as an optimal culture condition among other groups of the present study. Thus, the immunocytochemistry was done in SCB, 3 μM RA+Co-C (the selected group) and STO Co-C (control for selected group) groups.

Enrichment of mouse ESCs-derived PGCs was assessed using Mvh immunoreactivity [34]. The data obtained from the negative control showed no immunoreactivity to Mvh. The colour of the Mvh immunoreactive cells was green, which were either fibroblast-like or round (Figure 2). The mean percentage of the immunoreactive cells was evaluated and presented in Table 3. The level of Mvh was increased in both 3 μM RA+Co-C and STO Co-C groups relative to SCB group. The highest mean percentage of Mvh immunoreactive cells in 3 μM+Co-C and Co-C group was noticed in a way that the differences between 3 μM RA+Co-C group and the rest (SCB and STO Co-C groups) were significant (*P*<0.05), whereas the increased expression of this marker in STO Co-C group showed no significant difference with other groups (Table 3).

**Figure 2:** Cytochemistry of Mvh and CDH1 Positive immunostaining and negative controls for (**A**) Mvh marker characterizing the transdifferentiated PGCs (counterstained with ethidium bromide) and for (**B**) CDH1 marker used for characterizing the late germ cell differentiation. The cells immunostained with anti-Mvh and anti-CDH1 (arrow) antibodies that reacted with FITC-conjugated secondary antibodies in the STO Co-C and 3 μM RA concentrations+STO Co-C groups (×200) after 4 days induction with BMP4 followed by 7 days exposure with RA. The right panels show the phase contrast of the positive immunostained cells and negative control.

**Table 3:** The percentage of Mvh and CDH1 immunoreactive cells in the simple culture with BMP4 (SCB), STO Co-C and 3 μM RA concentrations+STO Co-C groups ^a^demonstrates significant difference with SCB and STO Co-C groups and ^b^shows significant difference with SCB group in the same rows (*P*≤0.05).

Markers	SCB	STO Co-C	3 μM RA+Co-C
Mvh	21.57±3.02	22.05±0.052	32.38±6.07^a^
CDH1	13.44±2.79	23.52±0.01^b^	32.8±6.3^b^

The result of immunocytochemistry of ESCs-derived PGCs differentiation into spermatogonial stem cells (SCCs) was assessed by CDH1, which were used as late premiotic germ cell marker (Figure 2) [35]. The CDH1 immunoreactive cells were counted like Mvh. In Table 3, the percentages of the CDH1 immunoreactive cells are shown. An increased level of late germ cell differentiation marker expression was observed in 3 μM+Co-C and STO Co-C groups compared with SCB group (*P*>0.05). The increase in CDH1 positive cells in 3 μM RA+Co-C and Co-C groups was significantly different with SCB group (*P*>0.05, Table 3).

## DISCUSSION

PGCs are the founder cells of germ cell lineage, and can be differentiated and proliferated in an induced system *in vitro* from stem cells. Thus, the enrichment conditions need to be optimized for improving the proliferation efficiency. In the present study, we demonstrated that the addition of 3 μM RA on the top of the STO feeder layer cells improved the proliferation of ESCs-derived PGCs.

Characterization of PGCs development is likely to lead to a better understanding of this important lineage. Advances in PGC isolation from 8.5 to 13.5 days old embryo and culture of these cells in different culture systems provide the opportunity to study the effect of different factors on the viability and proliferation of PGCs [36,37]. Primary experiments showed that culture medium conditioned by 10.5 dpc genital ridges caused an increase in the number of PGCs [38]. This matter leads to study for purification of factors *in vivo* with similar effects. To date, several growth factors with proliferative effects on PGCs *in vitro* have been known. An important implication that arises from culture of PGCs derived from epiblast *in vitro* is an increase in the number of these cells in response to signals such as FK, bFGF, LIF, stem cell factor (SCF), MGF, TNF-α, RA, BRL-CM and KL [20,21].

Our quantitative PCR data showed a higher ratio of Mvh expression, the PGC-specific marker [39,40], in 3 μM RA+Co-C group than others. Also, the immunocytochemistry results showed that the percentage of Mvh immunoreactive cells was higher in 3 μM RA+Co-C group than in STO Co-C group, indicating that the employment of 3 μM RA and STO as feeder have an apparent effect on PGC enrichment. These results confirmed those of previous investigations, which showed that RA and feeder layer was specifically required for PGC proliferation [15,16,19,21,23–26,31].

Koshimizu et al. [21] reported that intracellular signals induced by RA have an important role in PGC proliferation. It was also reported that addition of RA to PGCs derived from human bone marrow stem cell in culture caused the proliferation of PGCs [41]. The proliferative function of this factor may happen through shortening of cell cycle or induction of antiapoptotic signals in PGCs [42].

Also, it is reported that PGCs isolated from 8.5 to 10.5 days old embryo can continue to survive and proliferate *in vitro* when cultured on confluent monolayers of mouse feeder cells, either the bone marrow-derived cell line SI220 [19], the embryo fibroblast-derived cell line STO [23] or the Sertoli cells-derived cell line TM4 [16]. In another investigation, Co-C of human ESCs-derived PGCs with mouse fibroblast feeder layer cells was shown to have an apparent effect on PGCs enrichment [43].

PGCs survival and proliferation is supported by the feeder layer cells probably because these cells produce LIF and membrane-associated SCF as well as other factors that have not yet been characterized [17–19].

Furthermore, positive results achieved from *in vitro* culture of human PGCs isolated from 7 to 8 weeks old embryos on top of the fibroblast feeder layer cells in the presence of FK and KL [24–26]. These findings are consistent with the results of this investigation that indicates the RA and STO feeder layer roles in PGC enrichment.

In particular, it will be necessary to develop conditions that allow PGC proliferation without concomitant differentiation. For this purpose, the expression of Stra8, the specific marker for spermatogonia [44], was assessed. It was observed that 3 μM RA+Co-C conditions had no apparent effect on spermatogonial emergence.

CDH1 (previously known as E-cadherin), a marker for late premiotic germ cell [35], was assessed as well. No significant differences were noticed in 3 μM RA+Co-C and STO Co-C groups with each other and with SCB group. Tokuda et al. [35] reported that CDH1 is expressed specifically in undifferentiated type-A spermatogonia of mouse testis. Our results demonstrated that fewer cells tended to express CDH1, indicating that the majority of the cells transdifferentiated into germ cells were PGC.

In general, the maximum gene expression of Mvh, the PGC specific marker, was seen in the 3 μM RA+Co-C group. Also, the inductive effects were investigated immunocytochemically with Mvh and CDH1 antibodies. Immunocytochemistry results showed higher expression of Mvh in 3 μM RA concentrations on the top of the STO feeder layer. Meanwhile, assessment of the *Stra8* mRNA and CDH1 protein, the specific makers for spermatogonia, showed no significant differences between groups. As 3 μM RA+Co-C group had no negative effects on cell viability relative to control group and based on the immunocytochemistry/PCR results of PGC and spermatogonial markers, this group was selected as the best group among the mentioned groups of the present study.

## Abbreviations

bFGF: basic fibroblast growth factor
BMP4: bone morphogenetic protein-4
BRL-CM: buffalo rat liver cells
CCE: CCE is a mouse embryonic stem cell line derived from the 129/Sv mouse strain
CDH1: cadherin1
Co-C: co-culture
DEPC: diethylpyrocarbonate
DMEM: Dulbecco's modified Eagle's medium
dNTP: deoxynucleotide
EB: embryoid body
ESC: embryonic stem cell
FK: forskolin
KL: kit ligand
LIF: leukaemia inhibitory factor
MGF: macrophage growth factor
Mvh: mouse vasa homologue
PGC: primordial germ cell
Piwil2: piwi (Drosophila)-like 2
RA: retinoic acid
SCB: simple culture with BMP4
SCF: stem cell factor
STO: SIM mouse embryo-derived thioguanine- and ouabain-resistant
Stra8: stimulated by retinoic acid 8
TGF-b: transforming growth factor beta
TM4: an established cell line
TNF: tumour necrosis factor
VASA: mouse vasa homologue
